The article "Baseline neutrophilia, derived neutrophil‐to‐lymphocyte ratio (dNLR), platelet‐to‐lymphocyte ratio (PLR), and outcome in non small cell lung cancer (NSCLC) treated with Nivolumab or Docetaxel" was published in 2018. Journal: J Cell Physiol.

# Baseline neutrophilia, derived neutrophil‐to‐lymphocyte ratio (dNLR), platelet‐to‐lymphocyte ratio (PLR), and outcome in non small cell lung cancer (NSCLC) treated with Nivolumab or Docetaxel

**DOI:** 10.1002/jcp.26609

**Published:** 2018-04-19

**Authors:** Alessandro Russo, Tindara Franchina, Giuseppina R.R. Ricciardi, Alessandra Battaglia, Antonino Scimone, Rosa Berenato, Antonio Giordano, Vincenzo Adamo

**Affiliations:** ^1^ Medical Oncology Unit A.O. Papardo & Department of Human Pathology University of Messina Messina Italy; ^2^ Department of Medicine, Surgery and Neuroscience University of Siena and Istituto Toscano Tumori (ITT) Siena Italy; ^3^ Sbarro Institute for Cancer Research and Molecular Medicine, Center for Biotechnology, College of Science and Technology Temple University Philadelphia Pennsylvania

**Keywords:** biomarker, neutrophil‐to‐lymphocyte ratio, Nivolumab, NSCLC, platelet‐to‐lymphocyte ratio

## Abstract

Nivolumab is a novel therapeutic option in NSCLC, associated with a significant survival gain compared with Docetaxel. However, predictive biomarkers are lacking. The presence of systemic inflammation has been correlated with poor outcome in many cancer types. We aimed to evaluate whether there is a correlation between some indicators of inflammation and response to Nivolumab or Docetaxel in pre‐treated NSCLCs. Data of 62 patients receiving Nivolumab or Docetaxel were analyzed. Baseline neutrophilia and thrombocytosis were not associated with response. High dNLR was associated with no response to Nivolumab, but not with Docetaxel, whereas high PLR correlated with low treatment response in both groups. Among refractory patients, a higher incidence of thrombocytosis, neutrophilia, high PLR, and high dNLR levels were observed compared with the overall population. This is one of the first reports in this field and suggests that indicators of inflammation might be included together with other predictive biomarkers in the baseline evaluation of patients candidate for immunotherapy.

## 1 INTRODUCTION

Nivolumab is a novel therapeutic option in 2nd line Non Small Cell Lung Cancer (NSCLC) with both squamous and non‐squamous histology (Paz‐Ares, Horn, Spigel, Steins, & Ready, 2015; Reckamp, Baas, Crinò, Eberhardt, & Poddubskaya, 2015). However, predictive biomarkers are lacking. PD‐L1 IHC expression has been extensively studied in NSCLC as potential predictive biomarker of response to anti‐PD1/PD‐L1 agents with contrasting results and is now adopted as selection criteria for Pembrolizumab in both 1st and 2nd line therapy (Herbst et al., 2016; Reck et al., 2016).

Tumor‐promoting inflammation is an established hallmark of cancer, as chronic inflammation is a consistent feature of tumor microenvironment (Galdiero, Garlanda, Jaillon, Marone, & Mantovani, 2013; Hanahan & Weinberg. 2011). In addition, the presence of systemic inflammation correlates with poor outcome in many cancer types, including NSCLC. The immune cell composition of NSCLC is dominated by neutrophils (Kargl et al., 2017) and recently several authors correlated the presence of high neutrophil‐to‐lymphocyte ratio (NLR) and/or high absolute neutrophil count (ANC) with poor prognosis and lower response to conventional treatments in NSCLC (Carus et al., 2013; Derman et al., 2017; Kang et al., 2017; Scilla et al., 2017). Similar findings were reported for high platelet‐to‐lymphocyte ratio (PLR) (Gu et al., 2016; Sanchez‐Salcedo et al., 2016).

The article "Baseline neutrophilia, derived neutrophil‐to‐lymphocyte ratio (dNLR), platelet‐to‐lymphocyte ratio (PLR), and outcome in non small cell lung cancer (NSCLC) treated with Nivolumab or Docetaxel" was published in 2018. Journal: J Cell Physiol.

We aimed to evaluate whether there is a correlation between some indicators of inflammation status, including neutrophilia, high NRL, and high PLR with response in pretreated NSCLC patients receiving Nivolumab or Docetaxel.

## 2 MATERIALS AND METHODS

In this retrospective monocentric study twenty‐eight consecutive patients with NSCLC receiving Nivolumab were included. Baseline white cell count (WBC) and absolute neutrophil count (ANC) were collected and correlated with tumor response. Thirty‐four NSCLC patients treated with Docetaxel were used as controls. An ANC ≥7500 cell/μl was defined as neutrophilia. Derived neutrophil‐to‐lymphocyte ratio (dNLR) was calculated as: ANC/(WBC‐ANC). Platelet‐to‐lymphocyte ratio (PLR) was defined as platelet count (PLT)/lymphocyte count. dNLR ≥3 and PLR ≥160 were defined high. PLT ≥450 × 103/µl was defined as thrombocytosis (Ferrucci et al., 2016; Kim et al., 2016). Categorical variables were compared using chi‐square or Fisher's exact test. Overall survival (OS) was defined as time from Nivolumab or Docetaxel start to death and Progression Free Survival (PFS) as time from treatment start to Progression Disease (PD) or death for any cause. OS and PFS survival were estimated using the Kaplan–Meier method. Survival curves were compared using the log‐rank test. To estimate the hazard ratio (HR), Cox regression analysis was used. Statistical analyses were performed with the R program version 3.3.2.

## 3 RESULTS

Baseline characteristics of patients in our cohort are reassumed in Table 1. In the study population, median age was 68 years (range 45–82), 77% were male (89.3% in the Nivolumab group vs. 67.7% in the Docetaxel group, *p =* 0.0004) and the predominant histology was adenocarcinoma (48%), followed by squamous (40%), and mixed/other histotypes (12%). Most patients were current or former smokers (90%) with an equal distribution between the subgroups (*p =* 0.3572). Among non‐squamous patients, 16.2% were EGFR mutated and 8.1% were KRAS‐mutated, with an equal distribution in both treatment groups (*p = *0.0649 for EGFR mutations and *p = *0.9188 for KRAS mutations). The majority of patients received Nivolumab or Docetaxel as second line therapy (69.3%), with no statistical differences between subgroups (*p =* 0.205).

The article "Baseline neutrophilia, derived neutrophil‐to‐lymphocyte ratio (dNLR), platelet‐to‐lymphocyte ratio (PLR), and outcome in non small cell lung cancer (NSCLC) treated with Nivolumab or Docetaxel" was published in 2018. Journal: J Cell Physiol.

**Table 1:** Baseline characteristics of patients in our cohort

	All (62 patients)	Nivolumab (28 patients)	Docetaxel (34 patients)	*p* value
Median age	68 years (45‐82)	69 years (47‐78)	68 years (45‐82)	0.9315
Sex				0.0004
Male	77%	89.3%	67.7%	
Female	23%	10.7%	32.3%	
Smoking status				0.3572
Former/current smokers	90%	93%	88.2%	
Never smokers	10%	7%	11.8%	
Histology				
Squamous	40%	60.8%	23.5%	<0.0002
Adenocarcinoma	48%	39.2%	55.9%	0.0262
Mixed histology/other	12%	0%	20.6%	<0.0005
Biomolecular status (non‐SqCC only)				
EGFR‐mutated	16.2%	9.1%	19.2%	0.0649
EGFR wild‐type	83.8%	90.9%	80.8%	0.0649
KRAS mutated	8.1%	9.1%	7.7%	0.9188
Treatment lines				0.205
2nd line	69.3%	64.2%	73.5%	
≥3 lines	30.7%	35.8%	26.5%	

The overall response rate (ORR) in the study population, according to RECIST 1.1, was 12.5% with Nivolumab versus 9.0% with Docetaxel (*p =* 0.568); moreover, 8.3% of patients treated with Nivolumab experienced unconventional responses.

ORRs according to baseline inflammation markers are reassumed in Table 2. Baseline neutrophilia was detected in 18% and 26% of patients in the Nivolumab and Docetaxel subgroups, respectively, and thrombocytosis was found in 3.5% and 3% of patients, respectively. Baseline neutrophilia and thrombocytosis were associated with a significant reduction in the probability of response both in the global study population (*p* *= *0.0003 and *p* *= *0.0018, respectively) and in Nivolumab (*p* *= *0.0001 and *p* *= *0.0004, respectively) and Docetaxel (*p* *= *0.0006 and *p* *= *0.0042, respectively) subgroups. High dNLR was associated with lower ORRs with Nivolumab (*p* *= *0.0001), whereas no statistically significant differences were observed in the total study population (*p* *= *0.0787) and in patients treated with Docetaxel (*p* *= *0.9319). Conversely, a high PLR predicted a poor response in the overall study population (*p* = 0.0407) and in the two treatment subgroups (*p < *0.0004 and *p* *= *0.0094 for Nivolumab and Docetaxel, respectively).

**Table 2:** Overall response rates (ORRs) according to baseline dNLR, PLR, neutrophilia, and thrombocytosis in the total study population and in treatment subgroups

	High dNLR (%)	Low dNLR (%)	*p* value
ORR in the total population	5.26	13.51	*p *= 0.0787
ORR in the Nivolumab subgroup	0	15.78	*p *= 0.0001
ORR in the Docetaxel subgroup	12.5	11.11	*p *= 0.9319
	**High PLR (%)**	**Low PLR (%)**	**p value**
ORR in the total population	4.35	13.63	*p* = 0.0407
ORR in the Nivolumab subgroup	8.3	46.15	*p* < 0.0004
ORR in the Docetaxel subgroup	0	8.33	*p* = 0.0094
	**Neutrophilia (%)**	**No neutrophilia (%)**	***p* value**
ORR in the total population	0	14.28	*p* = 0.0003
ORR in the Nivolumab subgroup	0	15.78	*p* = 0.0001
ORR in the Docetaxel subgroup	0	13.04	*p* = 0.0006
	**Thrombocytosis (%)**	**No thrombocytosis (%)**	***p* value**
ORR in the total population	0	11.11	*p* = 0.0018
ORR in the Nivolumab subgroup	0	13.63	*p* = 0.0004
ORR in the Docetaxel subgroup	0	9.68	*p* = 0.0042

Moreover, we analyzed the baseline characteristics of refractory patients (i.e., progressive disease as best response) compared with the global study population. We found a higher incidence of thrombocytosis (7% and 5%, *p* *= *0.765), neutrophilia (28.5% and 40%, *p* *= *0.117), high PLR (75% and 50%, *p* *= *0.0004), and high dNLR levels (28.5% and 55%, *p* *= *0.0002) in this poor prognosis subgroup compared with the overall cohort of patients.

The article "Baseline neutrophilia, derived neutrophil‐to‐lymphocyte ratio (dNLR), platelet‐to‐lymphocyte ratio (PLR), and outcome in non small cell lung cancer (NSCLC) treated with Nivolumab or Docetaxel" was published in 2018. Journal: J Cell Physiol.

After a median follow‐up of 17.0 months (range 3–58), median PFS in the study population was 4.0 months with Nivolumab (CI 95%, 2.0‐NA), corresponding to a 6‐month PFS rate of 40% (CI 95%, 25–65), and 2.0 months with Docetaxel (CI 95%, 2.0–5.0), corresponding to a 6‐month PFS rate of 23.5% (CI 95%, 13–43). This difference was not statistically significant (*p* *= *0.0934; HR 0.64). Patients with no baseline neutrophilia tended to have longer PFS than those with neutrophilia in the whole study population (4.0 vs. 2.0 months; *p* *= *0.223) (Figure 1a) and in both Nivolumab (6.0 vs. 1.0 months; *p* *= *0.209) and Docetaxel (3.0 vs. 2.0 months; *p* *= *0.003) subgroups (Figures 1b and 1c).

**Figure 1:** Kaplan–Meier curves for PFS and OS according to the absolute neutrophil count (ANC) levels. (a) PFS in the study population; (b) PFS in the Nivolumab subgroup; (c) PFS in the Docetaxel subgroup; (d) OS in the study population; (e) OS in the Nivolumab subgroup; (f) OS in the Docetaxel subgroup

Patients with high and low dNLR experienced similar PFS (2.5 vs. 3.0 months; *p* *= *0.19) in the global study population (Figure 2a), as well as in patients treated with Nivolumab (1.0 vs. 4.0 months; *p* *= *0.924) (Figure 2b), and Docetaxel (2.5 vs. 3.0 months; *p* = 0.204) (Figure 2c). A high PLR (≥160) predicted a poor PFS (2.0 vs. 5.0 months) (Figure 3a), albeit this difference was not statistically significant (*p =* 0.172). No differences were reported when analyzing the two treatment subgroups with Nivolumab (6.0 vs. 6.0 months, *p =* 0.437) and Docetaxel (3.0 vs. 3.0, *p =* 0.961). Median OS in the study population was 5.0 months (CI 95%, 3–12) with Docetaxel and 6.0 months with Nivolumab (CI 95%, 3‐NA), with no statistical significant differences (*p = *0.456; HR 0.81). High dNLR predicted a poor OS in both overall population (3.5 vs. 9.0 months; *p =* 0.05) (Figure 2d) and with Nivolumab (2.0 vs. 6.0 months, *p = *0.789) (Figure 2e) and Docetaxel (3.5 vs. 8.5 months, *p = *0.071) (Figure 2f). Moreover, neutrophilia predicted a poorer OS in all patients (2.0 vs. 9.0 months, *p =* 0.005) (Figure 1d) and also in the Nivolumab (2.0 vs. 9.0 months, *p =* 0.245) (Figure 1e) and Docetaxel (2.0 vs. 8.0 months, *p =* 0.003) (Figure 1f) subgroups.

The article "Baseline neutrophilia, derived neutrophil‐to‐lymphocyte ratio (dNLR), platelet‐to‐lymphocyte ratio (PLR), and outcome in non small cell lung cancer (NSCLC) treated with Nivolumab or Docetaxel" was published in 2018. Journal: J Cell Physiol.

**Figure 2:** Kaplan–Meier curves for PFS and OS according to the derived neutrophil‐to‐lymphocyte ratio (dNLR). (a) PFS in the study population; (b) PFS in the Nivolumab subgroup; (c) PFS in the Docetaxel subgroup; (d) OS in the study population; (e) OS in the Nivolumab subgroup; (f) OS in the Docetaxel subgroup

**Figure 3:** PFS and OS curves according to platelet‐to‐lymphocyte ratio (PLR). (a) PFS in the study population and (b) OS in the study population with high PLR (≥160) or low PLR (<160)

Finally, patients with high PLR levels tended to have a shorter OS in the overall population (4.0 vs. 12.0 months, *p =* 0.085) (Figure 3b) and with both Nivolumab (6.0 vs. 10.0 months, *p* *= *0.756) and Docetaxel (4.0 vs. 8.5 months, *p = *0.352) compared to those with PLR levels <160, albeit these differences were not statistically significant.

## 4 DISCUSSION

Immune checkpoint inhibitors are rapidly re‐shaping the therapeutic landscape of NSCLC in both pre‐treated and chemotherapy naïve patients (Borghaei et al., 2015; Brahmer et al., 2015; Herbst et al., 2016; Reck et al., 2016; Rittmeyer et al., 2017) with unprecedented results in terms of overall survival. However, the advent of this innovative class of anticancer agents brings several novel challenges in clinical practice, such as new response criteria (Seymour et al., 2017), novel potential patterns of progression (Champiat et al., 2016), undeniable high costs (Matter‐Walstra et al., 2016), and most importantly the need of predictive biomarkers for patients selection. PD‐L1 immunohistochemical expression is the best‐studied predictive biomarker to anti‐PD1/PD‐L1 agents. However, the use of this biomarker for patient selection poses different biological and technical issues (Kerr et al., 2015; Patel & Kurzrock, 2015) and has produced contrasting results in clinical trials, with a significant proportion of patients responding to these agents even in absence of PD‐L1 expression (Borghaei et al., 2015; Brahmer et al., 2015; Rittmeyer et al., 2017). Several different predictive biomarkers beyond PD‐L1 IHC expression have been studied (Chen et al., 2016; Daud et al., 2016; Prat et al., 2017; Rizvi et al., 2015), but to date none has entered into clinics. Moreover, in some instances the clinical implementation of these methodologies is difficult due to high costs and high level of expertise required.

The article "Baseline neutrophilia, derived neutrophil‐to‐lymphocyte ratio (dNLR), platelet‐to‐lymphocyte ratio (PLR), and outcome in non small cell lung cancer (NSCLC) treated with Nivolumab or Docetaxel" was published in 2018. Journal: J Cell Physiol.

Inflammatory reaction results in chronic illnesses, including cancer (Rajendran et al., 2018). Inflammation is a hallmark of cancer and is a known driver of cancer development and progression. Different markers of inflammation have been investigated in NSCLC and other solid tumors and correlated with poor outcome and low therapeutic response. dNLR and PLR, in addition to neutrophilia and thrombocytosis are the most well‐studied markers of systemic inflammation in cancer and can be easily performed in clinical practice.

Tumor microenvironment and immune system play a central role in response to immunomodulating agents (Nishino, Ramaiya, Hatabu, & Hodi, 2017) and, recently, it has been reported that neutrophils dominate the immune cell composition in NSCLC (Kargl et al., 2017).

Here, we demonstrated that the presence of some indicators of systemic inflammation, such as baseline neutrophilia, thrombocytosis, high dNLR, and high PLR are associated with poor outcome in pre‐treated NSCLC and with low response to both Nivolumab and chemotherapy. These data confirm the poor prognostic role of these indicators in NSCLC, as previously reported (Akinci Ozyurek et al., 2017; Gu et al., 2016; Kang et al., 2017; Scilla et al., 2017). Moreover, recently, some authors have correlated high pre‐treatment dNLR and/or PLR levels with inferior outcomes in advanced NSCLC after treatment with Nivolumab (Bagley et al., 2017; Diem et al., 2017). These data are in line with our present analysis and suggest the utility of dNLR and PLR, besides other predictive biomarkers, for selection of patients to PD‐1/PD‐L1 axis inhibitors in NSCLC. In addition, we correlated the presence of baseline neutrophilia with outcome, demonstrating a negative predictive role in terms of PFS and OS in pre‐treated unselected NSCLCs with both chemotherapy and immunotherapy.

Our study presents some limitations. First, the retrospective nature of this analysis that may have introduced potential bias and confounding factors. However, in this monocentric study, were included all consecutive NSCLC patients treated with Nivolumab or Docetaxel, limiting the potential bias of selection inherited in this type of analyses. Second, the IHC status of PD‐L1 was available only in a minor fraction of patients, since it was not performed as routine clinical practice at the time of patients’ treatment, and was not included in the present analysis.

The article "Baseline neutrophilia, derived neutrophil‐to‐lymphocyte ratio (dNLR), platelet‐to‐lymphocyte ratio (PLR), and outcome in non small cell lung cancer (NSCLC) treated with Nivolumab or Docetaxel" was published in 2018. Journal: J Cell Physiol.

Future prospective studies, evaluating the role of these markers of systemic inflammation in addition to other predictive biomarkers will add further evidence of their potential role in the clinical decision making in NSCLC. The wider use of PD‐L1 testing after the approval of Pembrolizumab in PD‐L1+ ≥50% patients as first line treatment and in PD‐L1+ ≥1% patients in subsequent lines of therapy will facilitate the correlation of PD‐L1 status and markers of systemic inflammation with the outcome after anti‐PD1/PD‐L1 inhibitors.

## 5 CONCLUSIONS AND FUTURE PERSPECTIVES

The results of this study suggest that indicators of inflammation such as baseline neutrophilia, thrombocytosis, and high dNLR are usually associated with a dismal prognosis and low efficacy of both chemotherapy and immunotherapy in NSCLC. Given their relative easy estimation, baseline evaluation of these indicators may be included together with other predictive biomarkers in the baseline evaluation of patients candidate for immunotherapy.

## CONFLICTS OF INTEREST

No potential conflicts of interest declared.
